# Efficacy of Arthroscopic Meniscal Surgery Versus Conservative Management on Knee Pain and Functional Outcomes: A Meta-Analysis of Randomized Controlled Trials

**DOI:** 10.7759/cureus.74349

**Published:** 2024-11-24

**Authors:** Abdelfatah M Elsenosy, Ahmed Elnewishy, Radwa A Delewar

**Affiliations:** 1 Trauma and Orthopaedics, University Hospitals Dorset NHS Foundation Trust, Poole, GBR; 2 Trauma and Orthopaedics, Royal Berkshire Hospital, Reading, GBR; 3 Pharmacy, Alexandria University, Alexandria, EGY

**Keywords:** conservative management, degenerative meniscal tear, functional outcomes, knee pain, meniscal surgery, meta-analysis

## Abstract

Knee pain is a prevalent issue among older adults, often resulting from degenerative joint changes, and significantly impacts functionality and quality of life. While arthroscopic meniscal surgery is a common intervention for managing knee pain, its effectiveness compared to conservative treatments remains debated. This meta-analysis aims to compare the efficacy of arthroscopic meniscal surgery versus conservative management in alleviating knee pain and enhancing functional outcomes in patients with degenerative meniscal tears. We conducted a systematic review and meta-analysis of randomized controlled trials (RCTs) sourced from PubMed, Web of Science, and Scopus. The focus was on studies evaluating knee pain and function in patients aged 40 and older. Primary outcomes included knee pain reduction, measured using scales such as the Knee Injury and Osteoarthritis Outcome Score (KOOS), Visual Analog Scale (VAS), and Western Ontario and McMaster Universities Osteoarthritis Index (WOMAC), and functional improvement, assessed by scores like the Knee Injury and Osteoarthritis Outcome Score for Activities of Daily Living (KOOS ADL) and Lysholm Knee Scoring Scale (Lysholm). A random-effects model was employed to account for variability across studies, with heterogeneity quantified using I². Nine RCTs, encompassing a total of 1,200 patients, met the inclusion criteria. Pain outcomes indicated similar improvements in both the arthroscopic surgery and conservative management groups. The pooled standardized mean difference (SMD) for pain was -0.01 (95% CI: -0.36 to 0.34). Functional outcomes also showed minimal differences between treatments, with an SMD of -0.04 (95% CI: -0.21 to 0.13). Moderate heterogeneity (I²=70%) was observed, attributed to variations in conservative management protocols and patient characteristics across studies.

Arthroscopic meniscal surgery does not offer significant advantages over conservative management in reducing knee pain or improving function in patients with degenerative meniscal tears.

## Introduction and background

Knee pain is a common cause of functional impairment and disability among the elderly, often linked to knee osteoarthritis (OA) [1]. However, functional impairments are not inevitable with disease progression [2].

The rate of meniscal injuries has increased due to rising sports engagement and more degenerative tears. Arthroscopy is now the preferred treatment, even among older adults [3]. It is favored over open procedures for its smaller incision and quicker recovery [4,5]. Experts recommend it for mechanical symptoms when conservative treatments fail [6,7]. However, failure rates in patients over 40 range from 9% to 27% [8].

Success depends on factors like anterior knee laxity, tear location, patient age, lesion type, vascular zone involvement, time from injury to surgery, and surgeon skill [9]. Age impacts meniscal biology, with fewer meniscal cells in individuals over 40 [10].

Jaibaji et al. [10] found age affects meniscal cell density, with fewer cells in those over 40. The effectiveness of arthroscopic surgery versus conservative management remains debated [11-14].

This meta-analysis evaluates the efficacy of arthroscopic meniscal surgery compared to conservative management, focusing on clinical outcomes related to knee pain and function.

## Review

Methodology

Study Design

This meta-analysis adhered to established guidelines for the design, analysis, and reporting of meta-analyses [15]. Ethics committee approval was not required as this study involved only secondary analysis of published data without patient contact or identification.

Search Strategy

We conducted a comprehensive literature search using PubMed, Web of Science, and Scopus databases for relevant studies published up to September 2024. The search terms were tailored for maximum sensitivity in identifying studies comparing arthroscopic meniscal surgery and conservative management for knee pain and function outcomes. The following terms were used: "Arthroscopic meniscal surgery" AND "knee pain", "Meniscal repair" AND "conservative management", and "Meniscal injury" AND "functional outcomes". When applicable, Medical Subject Headings (MeSH) terms were utilized to enhance the search sensitivity.

Eligibility Criteria

Population: Adults (40 years and older) with meniscal tears associated with knee pain

Intervention: Arthroscopic meniscal surgery

Comparison: Conservative management (non-surgical interventions, including physical therapy and medications)

Outcomes: Primary outcomes focused on knee pain reduction (measured by the Knee Injury and Osteoarthritis Outcome Score (KOOS), Visual Analog Scale (VAS), Western Ontario and McMaster Universities Osteoarthritis Index (WOMAC), and Arthritis Impact Measurement Scales (AIMS)). Secondary outcomes included functional improvement (assessed by the Knee Injury and Osteoarthritis Outcome Score for Activities of Daily Living (KOOS ADL), Lysholm Knee Scoring Scale (Lysholm), Western Ontario and McMaster Universities Osteoarthritis Index (WOMAC), and Oxford Knee Score).

Study design: Randomized controlled trials (RCTs). Only studies published in English were included. Studies involving acute meniscal injuries without degenerative changes or patients below 40 years were excluded.

Screening and Data Extraction

EndNote (Clarivate, London, United Kingdom) was utilized to manage references and eliminate duplicate records. The initial screening was conducted by two independent reviewers based on titles and abstracts to exclude irrelevant studies. Full-text articles of potentially eligible studies were then assessed to ensure they met the inclusion criteria. Any disagreements between reviewers were resolved by consensus, and a third reviewer was involved to mediate unresolved discrepancies. Search results were summarized using a Preferred Reporting Items for Systematic Reviews and Meta-Analyses (PRISMA) flowchart to illustrate the selection process. Data extraction was conducted independently by two reviewers following a pre-specified data extraction form, which included study characteristics, patient demographics, and outcome measures. A third reviewer verified extracted data to maintain consistency and address any discrepancies.

Statistical Analysis

Statistical analysis was performed with the OpenMeta[Analyst] package for the meta-analysis. A grouped random-effects model was used to calculate the pooled mean outcome and create forest plots to display the individual study means of the two modalities to account for varying true effect sizes of the studies. A random-effects model was chosen to allow for the generalization of conclusions beyond the studies included in the analysis [16]. I^2^ was used to assess heterogeneity.

Results

Identification of the Studies

The initial search yielded 15 results, out of which six were excluded. This resulted in nine RCTs being included in the final quantitative synthesis (Figure 1). This meta-analysis focuses on evaluating the efficacy of arthroscopic meniscal surgery compared to conservative management, specifically targeting clinical outcomes related to knee pain and function. Key outcomes assessed include pain reduction, measured by various scales such as KOOS, VAS, WOMAC, and AIMS, and improvement in knee function, measured by KOOS ADL, Lysholm, WOMAC, and the Oxford Knee Score.

**Figure 1:** Flow diagram of the literature search and study selection processes

Quality Assessment of the Included Studies

The Cochrane Risk of Bias assessment chart visually demonstrates that the majority of the studies included in the analysis exhibit a low risk of bias across most domains, indicating a generally high quality of the included research (Figure 2). However, specific areas of concern were identified, notably in the studies by Chang et al. [17] and Vermesan et al. [18], which exhibited a moderate risk of bias in the "Random Sequence Generation" and "Blinding of Outcome Assessment" categories. Additionally, a few studies had unclear risks in categories like "Allocation Concealment" and "Other Biases". Despite these issues, the overall low risk of bias across most studies suggests that the findings of the meta-analysis are reliable, though the potential biases in the highlighted studies should be taken into consideration when interpreting the results.

**Figure 2:** Cochrane Risk of Bias assessment chart

Demographic Data

The demographic data of the included studies indicate that the average age of participants is generally around the mid-50s, with most studies reporting mean ages between 52 and 61 years. The gender distribution shows a slight male predominance in most studies, though some studies, such as Yim et al. [19], have a more balanced or female-skewed distribution. Sample sizes vary considerably, ranging from as few as 32 participants in Chang et al. [17] to as many as 330 participants in Katz et al. [20], with most studies including between 80 and 200 participants (Table 1).

**Table 1:** Demographic data of the included studies

Study	Year	Sample size (arthroscopic)	Sample size (conservative)	Age (years) (arthroscopic)	Age (years) (conservative)	Gender (M/F) (arthroscopic)	Gender (M/F) (conservative)
Gauffin et al. [21]	2017	75	75	54.0±5.0	54.0±6.0	53/22	56/19
Stensrud et al. [22]	2015	42	40	48.6±6.4	49.2±6.4	26/16	27/13
Vermesan et al. [18]	2013	60	60	59.2±7.5	57.6±7.8	-	-
Katz et al. [20]	2013	161	169	59.0±7.9	57.8±6.8	71/90	72/97
Herrlin et al. [23]	2013	47	49	54.0±5.0	56.0±5.8	28/19	30/19
Yim et al. [19]	2013	50	52	54.9±10.3	57.6±11.0	9/41	12/40
Kirkley et al. [24]	2008	92	86	58.6±10.2	60.6±9.9	38/54	28/58
Moseley et al. [25]	2002	120	60	52.4±11.4	52.0±11.1	111/9	56/4
Chang et al. [17]	1993	18	14	61.0±11.0	65.0±13.0	5/13	4/10

Pain Measurements

The pain measurement scores in the included studies reveal a range of outcomes across different follow-up periods and assessment tools. For example, KOOS pain scores at the final follow-up showed mean values such as 84.0±17.2 for arthroscopic surgery and 78.0±21.8 for conservative in Gauffin et al.'s study [21] over 36 months. In contrast, Herrlin et al. [23] reported scores of 94.5±14.9 and 100.0±15.1 over 60 months. Pain VAS scores in Yim et al.'s study [19] indicated similar pain relief levels after 24 months, with means around 1.8±1.0 for surgery and 1.7±0.8 for conservative management. WOMAC pain scores from Kirkley et al. [24] reported values of 168.0±134.0 for surgery and 185.0±132.0 for conservative treatment over 24 months. Finally, AIMS pain scores, as seen in Moseley et al. [25] and Chang et al. [17], also showed close results between the two treatment methods, with scores like 55.4±23.7 versus 52.5±25.1 in Moseley et al.'s study [25] after 24 months (Table 2).

**Table 2:** Pain measurement scores in the included studies KOOS: Knee Injury and Osteoarthritis Outcome Score; VAS: Visual Analog Scale; WOMAC: Western Ontario and McMaster Universities Osteoarthritis Index; AIMS: Arthritis Impact Measurement Scales

Pain measurement	Study	Pain at the final follow-up (arthroscopic)	Pain at the final follow-up (conservative)	End of follow-up
KOOS pain at the final follow-up	Gauffin et al. [21]	84.0±17.2	78.0±21.8	36 months
	Katz et al. [20]	19.1±17.8	19.3±17.9	12 months
	Herrlin et al. [23]	94.5±14.9	100.0±15.1	60 months
VAS pain at the final follow-up	Yim et al. [19]	1.8±1.0	1.7±0.8	24 months
WOMAC pain at the final follow-up	Kirkley et al. [24]	168.0±134.0	185.0±132.0	24 months
AIMS pain at the final follow-up	Moseley et al. [25]	55.4±23.7	52.5±25.1	24 months
	Chang et al. [17]	5.3	5.0	12 months

The forest plot in Figure 3 illustrates the standardized mean differences (SMD) in pain scores between arthroscopic meniscal surgery and conservative management groups across multiple RCTs. Each study presents its respective SMD with 95% confidence intervals (CI) to show the variation in pain outcomes based on the treatment type.

**Figure 3:** Forest plot of knee pain scores of randomized controlled trials between arthroscopic meniscal surgery and conservative management groups KOOS: Knee Injury and Osteoarthritis Outcome Score; VAS: Visual Analog Scale; WOMAC: Western Ontario and McMaster Universities Osteoarthritis Index; AIMS: Arthritis Impact Measurement Scales; SMD: standardized mean difference; SD: standard deviation; CI: confidence interval

Study-Specific Results

The KOOS pain scores reported by Gauffin et al. [21] show a slight trend favoring arthroscopic surgery with an SMD of 0.31, but the CI crosses zero, indicating that this difference is not statistically significant. Similarly, Herrlin et al.'s study [23] reports a negative SMD of -0.37, slightly favoring conservative management, though again, the CI crosses zero. Katz et al. [20] report an SMD of -0.01, showing virtually no difference between the groups. In the VAS pain scores, Yim et al. [19] found a small positive SMD of 0.11 favoring surgery, but with a CI crossing zero. The WOMAC pain scores from Kirkley et al. [24] indicate a slight favor towards conservative treatment with an SMD of -0.13, but this difference is also not statistically significant. Finally, the AIMS pain scores from Moseley et al. [25] and Chang et al. [17] show minimal differences between the groups, with SMD of 0.12 and 0.13, respectively, both of which have CI that cross zero.

Overall Effect

The pooled results under the random-effects model yield a combined SMD of -0.01, indicating no significant difference between arthroscopic surgery and conservative management in terms of pain relief. The CI (-0.36 to 0.34) also crosses zero, reinforcing the conclusion that there is no statistically significant difference in pain outcomes between the two treatment approaches.

Heterogeneity

The heterogeneity among the studies, as indicated by an I² of 70%, suggests moderate variability among the included trials. This level of heterogeneity reflects differences in patient populations, surgical techniques, conservative treatment protocols, and study designs, which contribute to the observed variation in pain outcomes.

Knee Function Measurement

The knee function measurement scores presented in Table 3 provide a detailed comparison of functional outcomes between arthroscopic surgery and conservative management across various studies. The KOOS ADL scores reported by Gauffin et al. [21] show comparable function outcomes at a 36-month follow-up, with mean scores of 87.0±15.0 for arthroscopic surgery and 82.0±20.1 for conservative management. The Lysholm scores from Herrlin et al. [23] and Yim et al. [19] indicate similar long-term functional outcomes, with Herrlin et al. [23] reporting slightly higher scores for conservative management after 60 months (95.0±3.8) compared to arthroscopic surgery (89.0±5.0), while Yim et al. [19] show minimal differences at 24 months. WOMAC function scores from Katz et al. [20] and Kirkley et al. [24] also reflect similar outcomes, with Katz et al. [20] showing almost identical scores after 12 months and Kirkley et al. [24] reporting slight variations at 24 months. The Oxford Knee Score from Vermesan et al. [18] presents a slight advantage for arthroscopic surgery with a score of 36.1±3.6 compared to 34.7±3.8 for conservative management after 12 months. Finally, AIMS function scores reported by Moseley et al. [25] and Chang et al. [17] suggest slight differences between the two treatment approaches, with Moseley et al. [25] showing slightly better function for surgery at 24 months and Chang et al. [17] reporting minimal differences at 12 months.

**Table 3:** Knee function measurement scores in the included studies KOOS ADL: Knee Injury and Osteoarthritis Outcome Score for Activities of Daily Living; Lysholm: Lysholm Knee Scoring Scale; WOMAC: Western Ontario and McMaster Universities Osteoarthritis Index; AIMS: Arthritis Impact Measurement Scales

Function scores at the final follow-up	Study	Arthroscopic surgery	Conservative management	Follow-up period
KOOS ADL	Gauffin et al. [21]	87.0±15.0	82.0±20.1	36 months
Lysholm	Herrlin et al. [23]	89.0±5.0	95.0±3.8	60 months
	Yim et al. [19]	83.2±12.0	84.3±10.5	24 months
WOMAC	Katz et al. [20]	13.7±16.2	14.5±16.3	12 months
	Kirkley et al. [24]	612.0±448.0	623.0±439.0	24 months
Oxford Knee Score	Vermesan et al. [18]	36.1±3.6	34.7±3.8	12 months
AIMS	Moseley et al. [25]	52.9±19.3	47.7±12.0	24 months
	Chang et al. [17]	1.7	2.0	12 months

The forest plot in Figure 4 illustrates the SMD in knee function scores between arthroscopic meniscal surgery and conservative management groups across several RCTs. Each study's SMD, along with its 95% CI, is presented to demonstrate the variability in functional outcomes based on the treatment type.

**Figure 4:** Forest plot of knee function scores of randomized controlled trials between arthroscopic meniscal surgery and conservative management groups KOOS ADL: Knee Injury and Osteoarthritis Outcome Score for Activities of Daily Living; WOMAC: Western Ontario and McMaster Universities Osteoarthritis Index; AIMS: Arthritis Impact Measurement Scales; SMD: standardized mean difference; SD: standard deviation; CI: confidence interval

Study-Specific Results

Gauffin et al.'s study [21], evaluating KOOS ADL function, shows a slight trend favoring arthroscopic surgery with an SMD of 0.28, although the CI crosses zero, suggesting no statistically significant difference. In the Lysholm function scores, Herrlin et al. [23] report a substantial negative SMD of -1.35, favoring conservative management, with a CI that does not cross zero, indicating a significant difference. Yim et al. [19] also report a small negative SMD of -0.10 in Lysholm scores, but with a CI that crosses zero, indicating no significant difference. The WOMAC function scores from Katz et al. [20] and Kirkley et al. [24] show SMD of -0.05 and -0.02, respectively, both with CI crossing zero, suggesting minimal differences between the treatment groups. The Oxford Knee Score from Vermesan et al. [18] indicates a slight favoring of arthroscopic surgery with an SMD of 0.38, which is statistically significant as the CI does not cross zero. Finally, AIMS function scores from Moseley et al. [25] and Chang et al. [17] indicate a slight trend towards better outcomes with arthroscopic surgery, with SMD of 0.30 and 0.13, but these are not statistically significant given the CI cross zero.

Overall Effect

The pooled results under the random-effects model suggest no significant overall difference in knee function between arthroscopic surgery and conservative management, with an SMD of -0.04 and a CI of -0.21 to 0.13. The CI crosses zero, indicating no statistically significant difference in function outcomes between the two groups.

Heterogeneity

The heterogeneity among the studies is high, particularly in the Lysholm and AIMS function scores, with I² values of 94% and 87%, respectively. This high level of heterogeneity indicates substantial variability across the studies, likely due to differences in study design, patient populations, surgical techniques, and conservative management protocols.

Discussion

This meta-analysis provides a comprehensive comparison between arthroscopic surgery and conservative management in terms of pain relief and knee function across various studies. The included studies utilized multiple outcome measures, such as KOOS, VAS, WOMAC, AIMS, Lysholm scores, and the Oxford Knee Score, allowing for a multidimensional assessment of both pain and functional outcomes. Despite the difference in patient populations, follow-up durations, and treatment protocols, the overall findings suggest minimal clinically significant differences between the two treatment approaches.

Although certain studies showed slight trends favoring one treatment over the other, the majority of the differences observed were not statistically significant. Additionally, the heterogeneity present in both pain and function outcomes, as indicated by high I² values in several subgroups, highlights the inherent variability across trials and suggests that patient characteristics and treatment protocols may play critical roles in influencing outcomes.

The results of this meta-analysis align with those reported in a systematic review that found the mean age of patients in the individual trials ranged from 52 and 61 years [26]. This age range is consistent with the typical onset of degenerative knee conditions, such as meniscal tears and osteoarthritis, which are more prevalent in middle-aged and older adults.

A meta-analysis by Snoeker et al. identified several risk factors for degenerative meniscal tears, including increased age, male sex, work-related kneeling and squatting, standing or walking >2 hours per day, walking >2 miles per day, climbing >30 flights of stairs per day, and lifting or carrying >10 kg >10 times per week. There was also some evidence suggesting that body mass index (BMI) >25 kg/m^2^ is a risk factor for degenerative tears, although too much heterogeneity between studies precluded the authors from conducting a meta-analysis. Sitting for >2 hours per day was shown to protect against degenerative tears. Risk factors for acute meniscal tears included playing soccer, rugby, and swimming; further, delayed anterior cruciate ligament (ACL) surgery (>12 months) was a risk factor for meniscal tears associated with knee laxity [27].

Several factors are risk factors for meniscal tears, increasing the likelihood of developing them. The non-modifiable risk factors for meniscal tears include sex, where the incidence in men is 2.5 times more than in women. Meniscal tears are more common in individuals with a biconcave tibial plateau and a discoid meniscus, those with lower extremity alignment issues, and those with ligamentous laxity. The modifiable risk factors that increase the risk of developing meniscal tears include a high BMI, certain occupations such as squatting, lifting and carrying weights, stair climbing, and sports-related activities, including football and rugby [27].

Our results also reveal that arthroscopic surgery offers minimal, short-term benefits in pain and function when compared to conservative management for degenerative knee disease, with no significant advantage over the long term. Various pain measurement tools and knee function scores across different studies show only marginal differences between the two treatment strategies, reflecting the limitations of arthroscopic surgery in providing meaningful, sustained improvements.

The systematic review and meta-analyses conducted on arthroscopic surgery for degenerative knee disease demonstrate that, while arthroscopic surgery may provide short-term relief in terms of pain and function, the long-term benefits compared to conservative management are negligible. The most prominent findings from high-quality meta-analyses confirm that conservative treatment offers comparable or superior long-term outcomes [13].

Multiple systematic reviews have examined the impact of arthroscopic surgery on pain relief in degenerative knee disease. A Cochrane review by Thorlund et al. compared the effectiveness of arthroscopic surgery to conservative treatments like physical therapy and found that there was only a small improvement in pain at three months post-surgery, but this difference was not clinically significant over the long term [13]. The review revealed that the SMD for pain was 0.14 at three months post-surgery, but after one year, there was no significant difference between surgery and conservative treatment [13].

Similarly, a systematic review by Khan et al. found that the improvement in pain scores from arthroscopy was not significant when compared to non-surgical management beyond six months of follow-up. The mean difference in pain scores using the VAS was minimal (0.06), and the CI suggested no substantial benefit from surgery [28].

When it comes to knee function, results from various systematic reviews and meta-analyses indicate little to no long-term benefit of arthroscopic surgery over conservative management. The Cochrane review by Thorlund et al. reported that, despite minor short-term improvements, the function scores using the WOMAC were not significantly better in the surgery group at the one-year follow-up. The SMD for function at 12 months was -0.11, favoring conservative management, but the difference was not clinically meaningful [13].

A broader meta-analysis by Brignardello-Petersen et al. emphasized the minimal long-term improvement in function between surgical and non-surgical approaches. Here, it was noted that while minor short-term improvements in function may occur post-surgery, they did not translate into long-term benefits, leaving conservative management as a highly effective option for patients with degenerative knee conditions [29].

One of the common challenges across these studies is the heterogeneity between patient populations, variations in surgical techniques, and differences in the definition of conservative management, which includes a wide range of interventions such as physiotherapy, pharmacotherapy, and activity modification. The meta-analysis by Brignardello-Petersen et al. [29] emphasized the issue of heterogeneity, noting an I² value of 89% across studies, indicating substantial variability that could affect the interpretation of pooled outcomes. Despite this, the overall conclusion remained that there were no clinically important differences in long-term outcomes between the two approaches.

Another review by Siemieniuk et al. focused on comparing knee arthroscopy with exercise-based therapies and highlighted that even though some studies reported short-term improvements in both pain and function, the long-term effects were negligible, with SMD for pain and function hovering around zero at 12 months This variability further underscores the need for individualized patient care, as the benefits of surgery appear to be limited and short-lived [30].

This meta-analysis' strength lies in its comprehensive coverage of high-quality RCTs, providing a robust comparison between arthroscopic surgery and conservative management. By focusing on large-scale studies and well-defined patient populations, the review offers clear evidence on the minimal benefits of surgery in the long term.

However, one limitation is the heterogeneity across studies in terms of follow-up duration, patient selection criteria, and the types of conservative management used. While most studies found no significant long-term differences between surgical and non-surgical approaches, the variation in conservative treatment protocols across studies introduces some uncertainty regarding the exact best practices for non-surgical management.

## Conclusions

This meta-analysis reveals no significant differences in pain relief or functional improvement between arthroscopic meniscal surgery and conservative management for patients over 40 with degenerative meniscal tears. Despite the prevalent use of arthroscopic surgery for symptomatic knee pain, the pooled SMD in pain and function scores across the included RCTs consistently demonstrated minimal benefit over conservative treatments. This is evidenced by overlapping confidence intervals and non-significant overall effect sizes.
